# Application of MRI and CT Images in Surgical Treatment of Early Cervical Cancer

**DOI:** 10.1155/2022/1592449

**Published:** 2022-08-02

**Authors:** An Lu, Guohua Lu

**Affiliations:** Obstetrics and Gynecology Department, Yixing City People's Hospital, Yixing, Jiangsu 214200, China

## Abstract

In order to understand the problems of the application of MRI and CT images in the early cervical cancer surgery, a method that the application of MRI imaging and CT images in early cervical cancer surgery was proposed. For the cervical cancer in clinical practice, the applications of the modern imaging examination and the clinical staging classification were investigated and analyzed. Compared with the surgical pathology results, the application value of common modern imaging in clinical staging of cervical cancer was evaluated. It was found that the sensitivity of MRI and CT in diagnosing lymph node metastasis was 56% and 58%, and the specificity was 93% and 92%, respectively. The experiment proved the application value of MRI and CT in clinical staging of cervical cancer.

## 1. Introduction

Since the 1940s, with the popularization of cervical cytology, HPV testing and other cervical cancer screening methods, patients with cervical cancer have been diagnosed and treated at the early stage or even precancerous stage, thus blocking the occurrence and development of cervical cancer. After the successful application of cervical cancer vaccine in clinic, the World Health Organization has put forward the ambitious goal of global elimination of cervical cancer. However, despite a significant decline in the incidence and mortality of cervical cancer in developed countries, cervical cancer is still one of the major malignant tumors threatening women's health worldwide, ranking fourth in the incidence and mortality of female malignant tumors, most of which occur in developing countries. In China, according to the tumor monitoring data of the National Cancer Center, cervical cancer ranks first among female reproductive tract malignancies. The prevention and treatment of cervical cancer is not only a simple medical issue but also affected by social, economic, cultural, and other complex factors in addition to medical factors. Research on the prevention and treatment of cervical cancer in China and other developing countries is not only necessary to reduce the imbalance in the prevention and treatment of cervical cancer, but also the only way to achieve the elimination of cervical cancer in the world.

## 2. Literature Review

Tuchina et al. believed that since tumor progression was a continuous process, patients with cervical cancer were presented as heterogeneous groups with different clinicopathological features and survival prognosis when they sought treatment [1]. Dong et al. believed that clinicians first judged patients' cancer stage and then conducted doctor-patient communication, prognosis judgment, and treatment plan selection according to their stages [2]. Therefore, Xiaodan et al. believed that accurate clinical staging was an important influencing factor in evaluating patient prognosis, selecting appropriate treatment mode, and implementing individualized surgery [3]. Low or high preoperative staging may lead to inadequate or excessive treatment of cervical cancer. Voronin et al. believed that the high staging caused some patients to lose the chance of surgery and accept direct radiotherapy instead, thus losing the advantages of surgical treatment in preserving ovarian and vaginal functions and reducing long-term complications. Some patients lost the opportunity to receive a smaller range of conservative surgery and received unnecessary extensive hysterectomy, resulting in increased perioperative complications and decreased quality of life [4]. Eley et al. believed that low staging could lead to inadequate treatment, and postoperative radiotherapy and chemotherapy were often needed, resulting in a significant increase in total complications and seriously affecting the quality of life. Or the scope of the lesion was found to be beyond the expectation during the operation, resulting in increased difficulty of the operation or even having to give up the operation [5]. In addition, Masselli et al. believed the clinical staging classification should be judged according to unified standards in patients with tumor staging, which could make the data of the world different medical institutions being comparable, so as to carry out data summary and analysis of therapeutic effect evaluation and the implementation of clinical trials. It could make cancer research results applied to the worldwide eventually [6]. Capozza et al. believed that cervical cancer was one of the earliest malignant tumors with clinical staging. Its history could be traced back to 1928 [7]. Reinhold et al. believed that the clinical staging classification was born in the context of radiotherapy as the main treatment for cervical cancer [8]. At that time, Marchenko et al. believed that in order to compare the therapeutic efficacy of cervical cancer among different institutions, different doctors, and different radiotherapy methods, a standard radiotherapy regimen for cervical cancer was established, which changed the chaotic situation of radiotherapy at that time. The following radiotherapy committee of the International Health Union commissioned three professors to develop clinical staging of cervical cancer [9]. After the staging was proposed, Silvestro et al. believed that it was gaining worldwide recognition because of its simplicity, practicality, and its ability to reflect prognosis to a certain extent. It was adopted by the Federation International of Gynecology and Obstetrics (FIGO) in 1954 and was used to today [10]. Although it was modified for many times, its periodization principle and framework remained unchanged. Compared with other malignant tumors using clinical staging, such as lung cancer, for a long time, the clinical staging of FIGO cervical cancer mainly relied on pelvic examination and some simple imaging methods, such as IVP and chest X-ray, while modern imaging examinations such as CT and MRI were excluded, as shown in Figure 1.

## 3. Methods

Full convolutional neural networks are widely used in image segmentation. At present, full convolutional neural network is used for organ segmentation in medical image. On the basis of full convolutional neural network, many improved network structures are derived. In the research, the basic structure and training method of convolutional neural network were introduced, and the three-dimensional convolutional neural network Vnet network was introduced, and then, the defects of Vnet network in the field of organ segmentation were pointed out. Full convolutional neural network is used to solve the problem of image semantic segmentation [11]. Since there is no full connection layer, the full convolutional neural network does not need to fix the feature graph into the feature vector of the same length, so it can receive the input image of any size. Full convolutional neural network is an end-to-end network structure, and the same size segmentation results can be obtained directly from the input image data. In essence, full-convolutional neural network classifies every pixel of the image [12, 13]. The full convolutional neural network is mainly composed of convolution layer, pooling layer, and upsampling layer. The function of convolution layer is to extract local features of image data. The function of pooling layer is to enhance receptive field and narrow data dimension. The function of the upsampling layer is to restore the feature map to the same size as the input image [14]. The overall process is as follows. The image is input first. Then, feature is extracted through convolution layer and pooling layer to compress feature dimension. Then, the dimension of the feature map is restored through the upper sampling layer. Finally, Softmax is calculated for the feature graph to obtain the category probability of each pixel. According to the probability, each pixel is classified and the final segmentation result is obtained. According to the dimension of input image, full-convolutional neural network can be divided into two-dimensional full-convolutional neural network and three-dimensional full-convolutional neural network. Common two-dimensional full convolutional neural network includes FCN, Unet, and DeepLab. Three-dimensional full convolutional neural network includes 3D Unet, Vnet, and DenseVnet. Full convolutional neural network is generally composed of the following parts including convolution, pooling, activation function, upsampling, and Softmax. Schematic diagram of the simple structure of full convolutional neural network is shown in Figure 2.

Pooling, namely, downsampling, is used to reduce data dimensions. Pooling typically reduces the dimension of the image data by a factor of 2. Due to the statistical properties of features, the feature graph can still describe the image after the pooling operation. And the pooling operation reduces the data dimensions, which can effectively avoid overfitting. There are three main types of pooling: maximum pooling, mean pooling, and convolution pooling. In maximum pooling, the maximum value of the region is selected as the output. In mean pooling, the mean value of the region is calculated as the output. In convolution pooling, the convolution is calculated, and the stride is set to 2 to achieve the effect of pooling [15]. After the input convolution calculation, another function will be applied, and this function is the activation function. The function of activation function is to introduce nonlinear relation so that the neural network can approximate to any nonlinear function.

Common activation functions are as follows.

Sigmoid function is shown in the following formula:

(1) $$\begin{array}{c} f\left(x\right)=\frac{1}{1+e^{-x}}. \end{array}$$

Hyperbolic tangent (tanh) function is shown in the following formula:

(2) $$\begin{array}{c} f\left(x\right)=\frac{e^{x}-e^{-x}}{e^{x}+e^{-x}}. \end{array}$$

ReLU function is shown in the following formula:

(3) $$\begin{array}{c} f\left(x\right)=\max\left(0,x\right). \end{array}$$

PReLU function is shown in the following formula:

(4) $$\begin{array}{c} f\left(y_{i}\right)=\left\{\begin{array}{c} y_{i},\text{if}y_{i}>0,\\ a_{i}y_{i},\text{if}y_{i}\leq 0. \end{array}\right. \end{array}$$

Sigmoid function is prone to cause the problem of gradient disappearance. Compared with sigmoid, tanh is improved but still has the problem of gradient disappearance. At the same time, these two functions are more complicated and require a large amount of calculation. ReLU function is greatly improved in these two aspects. ReLU not only does not appear gradient disappearance but also is easy to calculate. Meanwhile, ReLU function can also introduce sparsity into neural network. The PReLU function is unsaturated and converges faster than ReLU. After the convolution and pooling of the input image, the size of the feature map is smaller than the original image. The image segmentation network needs to restore the feature map to the same size as the input image for further calculation. Therefore, the size of the feature map needs to be expanded to improve the resolution of the feature map, which is called upsampling [16]. There are three common methods of upsampling: bilinear interpolation, transposed convolution, and antipooling. At present, transposed convolution is mainly used. Transposed convolution is performed by first enlarging the size of the input by adding zeros, then rotating the convolution kernel, and finally convolving the input. The operation is shown in Figure 3.

Softmax is used to deal with multiclassification problems. The final output of neural network needs to be processed by Softmax function. The definition of Softmax function is shown in the following formula:

(5) $$\begin{array}{c} s_{i}=\frac{e^{Vi}}{\sum_{i}^{c}e^{Vi}}. \end{array}$$

Full convolutional neural network is a supervised learning algorithm, and the parameters of the convolution kernel in the network need to be obtained through the supervised training. In the supervised training of convolutional neural network, three parts are mainly considered including labeled data, loss function, and gradient descent algorithm.

Loss function is used to measure the difference between the predicted value and the real value of the model. It is a nonnegative real value function. The smaller the loss function, the better the robustness of the model. For image segmentation, there are two commonly used loss functions.

Cross entropy loss function: it describes the difference between two probability distributions. The smaller the difference is, the closer the probability distribution is. For the two probability distributions *p* and *q*, *q* is used to represent the cross entropy of *p*, as shown in the following formula:

(6) $$\begin{array}{c} H\left(p,q\right)=-\underset{x}{\sum }P\left(x\right)\log q\left(x\right). \end{array}$$

Dice loss function: it describes the degree of overlap between the predicted region and the real region in the image segmentation result, as shown in the following formula:

(7) $$\begin{array}{c} D=\frac{2\sum_{i}^{N}p_{i}g_{i}}{\sum_{i}^{N}p_{i}^{2}+\sum_{i}^{N}g_{i}^{2}}. \end{array}$$

Gradient descent algorithm is a kind of iterative method. Gradient descent is one of the most commonly used methods for solving model parameters of machine learning algorithms, namely, unconstrained optimization problems. The minimum value of the target loss function was iteratively solved step by step by gradient descent method, and the minimum loss function and model parameter values were obtained. Commonly used gradient descent algorithms are as follows.

The full name of SGD is Stochastic Gradient Descent. A batch of samples are randomly selected. Each input in the sample is output by using the existing parameters, and then, all the errors are compared with the actual output. After averaging, the average error is obtained. Based on this, parameters are updated as shown in the following formulas:

(8) $$\begin{array}{c} \overset{\Lambda }{g}⟵+\frac{1}{m}\nabla_{\theta }\underset{i}{\sum }L\left(f\left(x_{i};\theta \right),y_{i}\right),\\ \theta ⟵\theta ‐\varepsilon \overset{\Lambda }{g}. \end{array}$$

One problem with SGD is that the gradient calculated in each iteration is noisy. Using the idea of momentum for reference, the previous several gradients are added into the calculation of this gradient, which can effectively alleviate the noise problem and speed up learning. The cumulative gradient decays each turn, as shown in the following formulas:

(9) $$\begin{array}{c} s⟵\rho_{1}s+\left(1-\rho_{1}\right)g,\\ r⟵\rho_{2}r+\left(1-\rho_{2}\right)g\Theta g. \end{array}$$

In the case of preparing the training data, the loss function and gradient descent algorithm are determined. Then, the full convolutional neural network can be trained to fit the parameter values of the neural network. However, the models trained based on training data sets often have poor generalization ability, which can be mainly divided into two reasons, namely, underfitting and overfitting. Underfitting is caused by the poor fitting degree of the model to the data, which can be solved by increasing the depth of the neural network or improving the network structure. Overfitting is because during the training of the model, if there is less training data, that is, the training data cannot estimate the distribution of the whole data or the number of training iterations is too many, the noise in the training data and the unrepresentative features in the training samples are fitted, which leads to the poor generalization ability of the model. The overall network structure is the encoder decoder structure. The left part is the encoding process, which is composed of convolution and pooling layer, with a total of 4 convolution layers and 4 pooling layers. The right part is decoding process, with a total of 4 convolution layers and 4 upsampling layers. In the middle of the network bottom is convolution layer, which is located between encoding and decoding process. In the encoding part and decoding part, the convolution layer with the same size of feature graph is connected by the cascade layer. Each convolution layer contains 1 to 2 convolution units, among which the first left convolution layer and the first right convolution layer contain 1 convolution unit, and the remaining convolution layers contain 2 convolution units. In the convolution layer, residual learning structure is adopted to add the input of the convolution layer and the final output of the convolution layer. And then, subsequent calculation is carried out, so as to alleviate the problem of gradient disappearance. The pooling layer of Vnet-S network is the convolution pooling. There are two 1 × 1 × 1 convolution kernels behind the right 1 convolution layer, which is responsible for the number of compression channels. At the end of the network is Softmax, which generates the category probability of each pixel of the image. Specific network parameters are shown in Table 1.

The overall process of network coding calculation is as follows. First, in the coding process, features are extracted continuously by the convolutional layer, feature dimensions are reduced by the pooling layer, and receptive fields are increased. When reaching the middle layer, feature dimensions reach the minimum and the number of feature channels reaches 256. Then, in the decoding process, the convolution layer extracts and combines the features, the upsampling layer restores the size of the feature image, and the cascade layer compensates the fine granularity image features and target location information. On the right 1, the size of the feature map of the convolution layer is restored to the same size as the input image. Then, two 1 × 1 × 1 convolution kernels are combined and the number of channels is compressed to obtain two feature images with the same size as the original image. Then, Softmax function is used to obtain the probability of each voxel in the original image belonging to foreground and background. If the foreground probability is greater than the background probability, the prediction is the foreground target and marked as 1. If the foreground probability is less than the background probability, the prediction is the background and marked 0. The loss function selected by training Vnet-S network is Dice loss function.

## 4. Experiment and Analysis

Twenty patients with LACC admitted to Nanfang Hospital of Southern Medical University from September 2020 to May 2021 were selected for a retrospective analysis. The original data sets of preoperative CTA and DSA images during arterial chemotherapy were collected. The patients were 29-52 years old, with an average age of 43.28 ± 7.98 years. All patients were evaluated by two chief gynecologic oncologists based on the 2009 Federation International of Gynecology and Obstetrics (FIGO) staging, and the size of the tumor was more than 4 cm. All patients were excluded from basic cardiovascular diseases, hyperthyroidism, pregnancy, etc., and had no history of drug or seafood allergy. After being informed of the efficacy and risks of arterial chemotherapy and other alternative treatment plans, they voluntarily accepted preoperative neoadjuvant arterial chemotherapy, underwent preoperative CTA examination, and signed relevant informed consent, as shown in Table 2.

Dual source CT (SOMATOM Definition) produced by Siemens, Uvixian (370 mgI/ml, Schering Guangzhou Pharmaceutical Co., LTD.) and double syringe were used. Scanning conditions were tube voltage 120 kV, tube current 320 mA, scanning layer thickness 5 mm, layer spacing 5 mm, fasting for 4 h to 6 h before examination, and without other special treatment. During the scanning, the patient was in supine position in the middle of the bed with his head in his hands and his legs straight and together. The midsagittal plane of his body was perpendicular to the bed. The scanning range was from the lower margin of the third lumbar spine to the lower margin of the symphysis pubis [17]. After the routine plain scanning was performed (plain scanning period), contrast agent 80 ml was injected through the patient's right median cubital vein at the flow rate of 4.0 m1/s (A tube) with a double simple high-pressure syringe, followed by 20 ml normal saline injection at 4.0 ml/s (B tube) and bolus tracking. The region of interest (ROI) at 2.0 cm above the abdominal aortic bifurcation was selected for dynamic CT value monitoring, and the scanning was automatically triggered when the CT value in ROI reached 100 Hu (arterial phase). Finally, the images of each period were thinned to a thickness of 1.0 mm and saved by disc carving. First, the original data set in plain scanning period was imported into the Mimics software. After automatic positioning images, tissue images, and interpolation processing, the minimum reconstruction threshold was set at 100 Hu. After region growing, a complete digital 3D model of pelvis was directly reconstructed. Finally, the constructed pelvic digital 3D model was exported and saved in STL format by binary STL command in export tool, in preparation for subsequent registration and reconstruction of vascular network model [18]. The original data set of arterial phase was imported into the Mimics software, and the minimum reconstruction threshold was set to 90 Hu~100 Hu according to the display of arterial blood network after automatic positioning image, tissue image, and interpolation processing. Then, the bone tissue of each layer was automatically generated, and the outline of arterial blood network was enhanced (initial mask) by region growth. The STL format file of pelvis was imported into the reconstruction file of arterial phase, and the 3D model data was inverted into 2D mask data by calculate mask from subject. After separating the pelvis from the connected part of the pelvic arterial network layer by layer, the pelvic mask was created by using erase tools in edit masks. Boolean operations were used to subtract the pelvic mask from the initial mask. A new digital 3D model of cervical cancer arterial blood network was further generated by using the region growth tool, which was exported and saved in JPEG format. On the basis of the digital 3D model of uterine arterial blood network for cervical cancer in vivo, 3Dview, Rotation, and Rescale were used to scale and rotate the model at any size and angle, so as to observe the branches and direction of each artery. The source and number of uterine blood supply arteries were identified. Using the function of Cut with polyplane and Cut with curve in the Mimics software, the uterine arterial blood network model was segmented into uterine or cervical arterial blood network, left or right uterine arterial blood network, and left or right cervical arterial blood network. For each part, the blood volume could be calculated by using 3D properties—volume and the blood supply ratio could be further calculated. For cervical cancer patients with original clinical IB1~IIA2 stage included in the research, lymph node metastasis was first determined according to MRI or CT examination reports. For patients with positive pelvic lymph nodes, IICr stage was defined according to the new FIGO cervical cancer staging standard. Since para-aortic lymph node dissection was performed in only a few cases, IIC stage in the research referred to the cases with positive pelvic lymph nodes. Then, according to the surgical pathological report, lymph node metastasis was determined, which was defined as IHICp stage in the same way. And then, IICr and IIICp were compared. The measurement data were expressed as mean ± standard deviation (*X* ± *S*), and the counting data were expressed as *N* (%). According to data type, intergroup comparison was performed by independent sample *t* test, and intergroup rate comparison was performed by *χ*^2^ test or Fisher's exact probability method. When lymph node metastasis was confirmed, it was defined as true positive if both MRI and pathological reports indicated the presence of at least one lymph node metastasis [19, 20]. If only MRI showed lymph node metastasis, it was defined as false positive. If neither MRI nor pathology showed lymph node metastasis, it was defined as true negative. If only pathology showed lymph node metastasis, it was defined as false negative. The sensitivity, specificity, positive predictive value, and negative predictive value of imaging examination in diagnosing lymph node metastasis were calculated using surgical pathological results as the gold standard. The SPSS 21.0 software was used for statistical analysis. A total of 46313 cases of cervical cancer were screened from the big database of clinical diagnosis and treatment of cervical cancer in China, and 6662 cases were selected for final analysis. The case screening process is shown in Figure 4.

With the gradual popularization of cervical cytology screening, HPV testing, and cervical cancer vaccine, there are great changes in the epidemiology of cervical cancer. Firstly, there are obvious national and regional differences [21]. In developed countries, cervical cancer on a whole has appeared a downward trend. But in the developing world, because of the disequilibrium of medical and health conditions, cervical cancer has not been effectively controlled. Even due to factors such as lifestyle changes, new cases continue to rise. Cervical cancer is still a serious threat to women's health gynecologic malignant tumor. Secondly, the wide application of cervical cancer screening makes more women get diagnosed at the early stage, and the diagnosis proportion of early cervical cancer increases. Thirdly, the incidence of cervical cancer shows an obvious trend of younger age. And patients often have the desire to preserve ovarian function or fertility. Finally, researches on the staging methods of cervical cancer show that in many countries worldwide, especially developed countries, the clinical staging of modern imaging examinations such as MRI is not strictly excluded but affected by these examinations [22]. The exclusion of modern imaging tests such as MRI from clinical staging is in fact not universally followed, leading to a decline in the comparability of clinical staging between different countries and regions worldwide. From the perspective of the change of treatment mode, with the increase of cases of early cervical cancer, the proportion of patients with cervical cancer undergoing surgical treatment is on the rise due to the advantages of surgical treatment in preserving ovarian function, tissue elasticity, and reproductive function [23]. Nowadays, the treatment mode of cervical cancer has changed into a comprehensive prevention and treatment mode. It is mainly diversified surgical treatments for early cancer and the radiotherapy combined with immunotherapy and gene therapy for middle and late cancer. Tumor staging is not static, but it should be regularly updated as clinical practice changes, so as to adapt to current clinical practice. Therefore, with the changes in the epidemiology and treatment mode of cervical cancer, the clinical staging of cervical cancer should be changed accordingly. For a long time, a large number of researches have believed that lymph node metastasis is an adverse factor affecting the prognosis of patients with early cervical cancer. The 5-year survival rate of patients with negative lymph node metastasis can reach 91%, while the 5-year survival rate of patients with positive lymph node metastasis decreases to 67%. Lymph node metastasis is also a determinant of postoperative supplementary radiotherapy. Therefore, in the new stage classification of cervical cancer, lymph node metastasis is included in the stage and defined as IIC stage. At the same time, modern imaging examinations such as MRI and CT are allowed to be included in the clinical stage, making it possible to assess the presence of lymph node metastasis through imaging examination before treatment. Since positive lymph nodes are one of the clear indications of postoperative supplementary radiotherapy, it is of great clinical significance to determine whether there is lymph node metastasis and whether it is IIC before treatment. On the one hand, if there is no actual lymph node metastasis and the imaging is determined to be stage IIC, the patient may be advised to direct radiation therapy, thus losing the opportunity for surgical treatment. For the women of childbearing age, radiotherapy may result in loss of ovarian function. And for the women who need to have children, radiotherapy may also result in loss of fertility. On the other hand, if positive lymph nodes are not found before surgical treatment, patients will need to receive supplementary radiotherapy after surgery, resulting in higher total complications of cervical cancer patients than direct radiotherapy and decreased quality of life [24, 25].

Therefore, if imaging methods can be used to accurately diagnose the presence of lymph node metastasis and improve the accuracy of IICr, it will certainly help improve the treatment prognosis of patients. At present, the accuracy of MRI and CT in diagnosing lymph node metastasis is not ideal. A meta-analysis showed that MRI and CT had a sensitivity of 56% and 58% and specificity of 93% and 92%, respectively, in diagnosing lymph node metastasis. Bourgioti et al. reported that MRI had a sensitivity of 50.00% and specificity of 98.99% in the diagnosis of positive pelvic lymph nodes. In the research, the sensitivity of MRI and CT in diagnosing lymph node metastasis was only 26.56% and 12.21%, respectively. Most patients with lymph node metastasis confirmed after surgery could not be accurately diagnosed by CT or MRI before surgery. The diagnostic efficacy of CT and MRI in diagnosing lymph nodes was not ideal. The reasons were analyzed, which may be related to the multicenter retrospective research, long time span, and the lack of advanced early imaging equipment. Therefore, in the clinical practice of cervical cancer in China, MRI and CT examination is used to diagnose lymph node metastasis, and the diagnostic efficacy of IIC stage is low [26]. Pelvic lymphatic dissection should still be considered for patients with cervical cancer whose MRI or CT examination does not indicate positive lymph nodes [27, 28]. Currently, the commonly used imaging techniques for detecting lymph node status in clinical practice include B-ultrasound, CT, MRI, and PET-CT. Among them, CT and MRI are the most commonly used imaging examinations for detecting lymph node status of cervical cancer due to their high popularity. MRI and CT are mainly used to judge benign and malignant lymph nodes by observing the size of lymph nodes, and the positive standard is usually shorter axis diameter ≥ 1 cm. However, normal-sized metastatic lymph nodes are not uncommon. And enlarged lymph nodes can also be benign lesions, such as inflammatory enlargement and reactive hyperplasia. Morphological criteria alone cannot distinguish whether the enlarged lymph nodes are metastatic lymph nodes and cannot distinguish inflammatory lesions from tumor metastasis. And normal size metastatic lymph nodes also cannot be found.

## 5. Conclusions

The application of FIGO clinical staging of cervical cancer in China was described in detail, including standardization and accuracy. The proportion of clinical staging not conforming to FIGO staging standard was 22.6%, and the nonstandard staging was more common in age > 70 years old. Nonexogenous lesions and other staging parameters were difficult to determine. The proportion of inaccurate clinical staging was 34.2%, and the incidence of higher stage was significantly higher than that of lower stage. The inconsistent judgment of tumor maximum diameter and vaginal involvement was the main factor leading to inaccurate staging classification. Imaging examination, such as MRI and CT, has application value in the clinical staging of cervical cancer. The inclusion of imaging examination in cervical cancer staging is helpful to improve the accuracy of clinical staging. In the past clinical practice of cervical cancer in China, the low diagnostic efficiency of imaging examination may be related to the relatively backward imaging examination equipment and technology and the insufficient attention of gynecological oncologists to imaging examination. MRI has the advantage of high soft tissue resolution, which can accurately display the size of cervical tumor lesions, especially suitable for early cervical cancer. CT scanning has the advantages of fast speed and clear images, which is more suitable for the late stage of cervical cancer.

## Figures and Tables

**Figure 1:** Application of MRI and CT images in the surgical treatment of early cervical cancer.

**Figure 2:** Schematic diagram of simple structure.

**Figure 3:** ROC comparison of different variables.

**Figure 4:** Case inclusion process.

**Table 1:** Vnet-S network parameters.

Convolution layer	Composition	Convolution layer	Composition
Left 1	Convolution unit X1 Channel number 16	Right 1	Convolution unit X2 Channel number 128
Left 2	Convolution unit X2 Channel number 32	Right 2	Convolution unit X2 Channel number 64
Left 3	Convolution unit X2 Channel number 64	Right 3	Convolution unit X2 Channel number 32
Left 4	Convolution unit X2 Channel number 128	Right 4	Convolution unit X1 Channel number 16
Middle layer	Convolution unit X2 Channel number 256	Output	1 × 1 × 1 convolution Channel number 2

**Table 2:** FIGO staging of cervical cancer patients.

Staging	Cases
IB2 stage	9 cases
IIA2 stage	3 cases
IIB stage	7 cases
IIIA stage	1 case
In total	20 cases

## Data Availability

The data used to support the findings of this study are available from the corresponding author upon request.
